The article "Knowledge, practice and associated factors of newborn care among postnatal mothers at health centers, Bahir Dar City, Northwestern Ethiopia, 2016" was retracted in 2020. Reasons: plagiarism; content taken from a thesis; overlap with other authors' work.

# Knowledge, practice and associated factors of newborn care among postnatal mothers at health centers, Bahir Dar City, Northwestern Ethiopia, 2016

**DOI:** 10.1186/s13104-019-4501-z

**Published:** 2019-08-05

**Authors:** Awoke Kebede

**Affiliations:** School of Nursing, College of Health Sciences and Comprehensive Specialized Hospital, Aksum University, Aksum, Ethiopia

**Keywords:** Newborn care, Practice, Knowledge, Mothers

## Abstract

**Objective:**

Most neonatal deaths occur in low income and middle-income countries and about half of the deaths occur at home. It is estimated that about 75% of neonatal deaths could be avoided with simple, low-cost tools that already exist such as antibiotics for pneumonia and sepsis, sterile blades to cut the umbilical cords using knit caps and kangaroo care to keep babies warm. The aim of this study is to assess the knowledge, attitudes, and practices of newborn care among postnatal mothers at Bahir Dar, Ethiopia 2016. An institutional based cross-sectional study design was used. The sample size was calculated by using a single population proportion formula. The total sample size was 422. The collected data was coded and entered to Epi-Data version 3.1 and exported and analyzed using SPSS version 23.0. Both descriptive and multivariate logistic regression was performed.

**Result:**

A total of 414 postnatal mothers were interviewed with a response rate of 98.1%, among them 55.3% had good knowledge and 60.6% had a good practice of newborn care. Age of the mother, occupation, the month of pregnancy at first ANC visits, overall knowledge and attitude level was found to have a significant association with newborn care practice.

## Introduction

Worldwide every year about 4 million die in the first 4 weeks of life. Most neonatal deaths occur in low and middle income countries and about half of the deaths occur at home. It is heartbreaking that millions of newborns die every year especially when their deaths are so easily preventable. It is estimated that about 75% of neonatal deaths could be avoided with simple, low-cost tools that already exist for example antibiotics for pneumonia and sepsis, sterile blades to cut the umbilical cords using knit caps and kangaroo care to keep babies warm [1–3].

Neonatal health and survival are improved by providing essential newborn care such as cleanliness, thermal protection, initiation of breathing, early and exclusive breastfeeding, eye care, immunization, and management of newborn illness [4–6]. Providing care of the children had always traditionally been the forte of mothers irrespective of education, income, and social class differences. The important task of motherhood is to fulfill physical, emotional, social, intellectual and moral needs of children. There is no qualm that a mother plays an important role in this regard [7].

The article "Knowledge, practice and associated factors of newborn care among postnatal mothers at health centers, Bahir Dar City, Northwestern Ethiopia, 2016" was retracted in 2020. Reasons: plagiarism; content taken from a thesis; overlap with other authors' work.

The maximum gap in newborn care is often during the critical first week of life when most neonatal and maternal deaths often occur at home and without any contact with the formal health sector. Some improper practices such as untrained attendants during delivery, unhealthy delivery practices, taboos and superstition associated with caring for the newborn greatly affect newborn survival. This study, therefore, required to identify the gaps in the knowledge and practices and associated factors mothers towards newborn care and to providing inputs into developing feasible and sustainable community-based interventions to improve neonatal survival.

## Main text

### The study area and period

The study was conducted in Public health centers of Bahir Dar City which are located in the 556 km away from Addis Ababa, the capital city of Ethiopia. The study was conducted from March 1–30, 2016.

### Study design

An institutional based Cross-sectional study design was conducted.

### Sample size

A total of 422 samples were calculated using a single population proportion formula by assuming 5% marginal error and 95% confidence interval (σ = 0.05) and by estimation of the proportion of Mothers’ knowledge and practice considering to be 50% and by adding 10% of non-response rate.

### Sampling method and sampling procedure

After allocating proportional to Postnatal care coverage of health centers, systematic random sampling methods from those found in all the healthcare facilities during data collection time was used until the sample size is fulfilled.

### Data collection instruments

#### Data collection tools

Data were collected by face to face interview using semi-structured questionnaires which are adopted from different kinds of literature [2–6] and include socio-demographic characteristic, knowledge and practice and factors associated with newborn care.

### Data collection technique

The data was collected by face to face interview using semi-structured questionnaires prepared in English and translated to local language Amharic. The supervisor and data collectors were assigned to follow the whole procedure of data collection after giving a brief description of the importance of the study and filled questionnaires were collected timely.

### Data quality control

The pre-test was done in 10% of the estimated sample size among nurses working in Dangla health center to evaluate the clarity; completeness and understandability of the questions in the questionnaire ensure the validity of instruments and reactions of the respondents to the questions on the study populations.

The article "Knowledge, practice and associated factors of newborn care among postnatal mothers at health centers, Bahir Dar City, Northwestern Ethiopia, 2016" was retracted in 2020. Reasons: plagiarism; content taken from a thesis; overlap with other authors' work.

### Data management and analysis of the result

Data was checked during data collection to ensure that all the information is properly collected and recorded. All the data was coded in terms of numbers and information was checked for completeness before and during data processing. After data collection, the response was coded and entered into Epi-Data version 3.1 software then it was exported to SPSS) version 23 software for analysis. P-value of < 0.05 and 95% confidence level was used as a difference of statistical significance. Finally, results were compiled and presented using tables, graphs, and texts.

### Ethical consideration

An Ethical Clearance was taken from an institutional review board of Aksum University College of health science and comprehensive specialized hospital. After explaining the purpose of the study, participant’s voluntariness was gained prior to their participation and they were informed that privacy and confidentiality were maintained. They were also informed that the study did not have any harm to them. Any nurse who is not willing to be included in the study was not being forced to include.

### Results

A total of 414 postnatal mothers were interviewed and the response rate was 98.1%. Most of the study participants 191 (46.1%) were in the age group of 25–29 years. Majority of respondents 355 (85.7%) were married, 291 (70.3%) were orthodox by religion, 220 (53.1%) were Amhara by ethnicity, 128 (30.9%) had Tertiary (> 12) education, 153 (37.0%) were a housewife.

Out of the total postnatal mothers interviewed, 401 (96.9%) had attended the antenatal clinic and from those postnatal mothers who had attended ANC clinic, 194 (46.9%) of them started their first visit at 3–6 month of gestation with an average of 3.48 visits. Majority of the mothers were primiparous 245 (59.2%). Almost all respondents 374 (90.3%) planed where to deliver their baby and 341 (82.4%) of newborns had a birth weight ranging 2.5–4 kilograms. Male neonates’ accounts 222 (53.6%) (Table 1).

**Table 1:** Distribution of socio-demographic characteristics of postnatal mothers in health centers, Bahir Dar, Ethiopia, 2016 (N = 414)

Variable	Category	Frequency	Percentage
Age of mother in years	15–19	11	2.7
	20–24	111	26.8
	25–29	191	46.1
	30–34	76	18.4
	35–39	25	6.0
Marital status	Single	49	11.8
	Married	355	85.8
	Divorced	10	2.4
Mother’s religion	Orthodox	291	70.3
	Catholic	13	3.1
	Protestant	62	15
	Muslim	48	11.6
Maternal educational level	Can’t read and write	45	10.9
	Read and write	29	7.0
	Primary (1–4)	29	7.0
	Primary (5–8)	70	16.9
	Secondary (9–12)	113	27.3
	Tertiary (> 12)	128	30.9
Occupation	House wife	153	37.0
	Private employee	114	27.5
	Government employee	101	24.4
	Merchant	35	8.5
	Student	11	2.6
Maternal monthly income	151–650	51	12.3
	651–1400	78	18.8
	1401–2350	133	32.2
	2351–3550	106	25.6
	3551–5000	33	8.0
	> 5000	13	3.1

Most of the respondents 330 (79.7%) were aware of the need fora newborn baby to be kept warm at birth. Majority of the respondents 275 (66.4%) replied time of newborns first bathing is after 1 day of birth and 76 (18.4%) of them said that newborn baby bathed immediately.

The article "Knowledge, practice and associated factors of newborn care among postnatal mothers at health centers, Bahir Dar City, Northwestern Ethiopia, 2016" was retracted in 2020. Reasons: plagiarism; content taken from a thesis; overlap with other authors' work.

Study subjects who knew about breastfeeding on demand (8 to 12 times per day), exclusive breastfeeding for 6 months, colostrum should be given to their newborns and optimal time of breastfeeding initiation is within 30–60 min’ accounts 114 (27.5%)/288 (69.6%), 372 (93.9%), 399 (96.4%) and 73 (17.6%) respectively. Majority 386 (93.2%) of the mothers knew that prelacteal feeds should not be given to neonates and 24 (5.8%) believed in giving their neonates. Almost all mothers 397 (95.9%) were aware of the need to vaccinate their newborns at birth while 374 (90.3%) knew that vaccines were given to prevent diseases. The overall knowledge score of the study participants shows that majority 229 (55.3%) of the respondents had good knowledge.

Regarding Cleanliness and cord care practice all mothers responded that baby was placed on the mother’s abdomen and a clean surface accounts 365 (88.2%) and 49 (11.8%) respectively before the placenta was expelled. The umbilical cord was cut with a new or boiled blade in 262 (63.3%) deliveries, and in 117 (28.3%) of them don’t know what was used. Most 404 (97.6%) replied as nothing was applied on the umbilical stump. But butter and Vaseline was applied in 10 (2.4%) of deliveries. The newborn was often wrapped in a new unwashed cloth 227 (54.8%) and 157 (37.9%) in an old washed cloth.

Concerning maintenance of warm chain for the newborn, all of the respondents were used either skin to skin or wrapped using a dry clean cloth to keep their baby warm. Majority of the respondents 204 (49.3%) said they bathed their newborn after 1 day of birth and 150 (36.2%) of them said that newborn baby bathed immediately.

Regarding breastfeeding almost all respondents 292 (70.58%) and 115 (27.8%) replied that as they feed their newborn 8 to 12 times and on-demand respectively. Almost all 406 (98.1%) newborns were breastfed and 397 (95.9%) newborns were initiated breastfeeding within an hour after delivery. The overall practice score of the study participants shows that majority 251 (60.6%) of the respondents had a good practice.

According to the result of multivariate analysis, only the mother ‘s level of education was significantly associated with their knowledge of newborn care; those respondents who completed primary (5–8) education were found to have 4.044 times more good knowledge about newborn care than those who had no formal education [AOR = 4.044, 95% CI (1.789, 9.142)] also with secondary (9–12) and tertiary (> 12) education, respondents were found to have 2.465 and 2.301 times more good knowledge about newborn care than those who had no formal education [AOR = 2.465, 95% CI (1.175, 5.173)] and [AOR = 2.301, 95% CI (1.114, 4.752)] (Table 2).

The article "Knowledge, practice and associated factors of newborn care among postnatal mothers at health centers, Bahir Dar City, Northwestern Ethiopia, 2016" was retracted in 2020. Reasons: plagiarism; content taken from a thesis; overlap with other authors' work.

**Table 2:** Association of knowledge on newborn care with socio-demographic and other factors, among postnatal mothers in Health Centers, Bahir Dar, Northwest Ethiopia, 2016 (N = 414)

Variable	Knowledge level				Odds ratio	
	Poor knowledge		Good knowledge		Crude	Adjusted
	N	%	N	%		
Maternal educational level						
No formal education	30	16.2	15	6.6	1	1
Read and Write	18	9.7	11	4.8	1.222 (0.462, 3.234)	1.362 (0.494, 3.753)
Primary (1–4)	12	6.5	17	7.4	2.833 (1.080, 7.433)*	2.679 (0.996, 7.205)
Primary (5–8)	21	11.4	49	21.4	4.667 (2.090, 6.421)*	4.44 (0.789, 9.142)
Secondary (9–12)	49	26.5	64	27.9	2.612 (1.268, 5.382)*	2.465 (1.175, 5.173)*
Tertiary (> 12)	55	29.7	73	31.9	2.655 (1.303, 5.409)*	2.301 (1.114, 4.752)*
Month of pregnancy at first ANC visit						
1–3 months	71	41.3	114	49.8	1	1
3–6 months	94	54.7	100	43.7	0.663 (0.440, 0.997)*	0.714 (0.466, 1.093)
6–9 months	7	4.0	15	6.5	1.335 (0.519, 3.433)	1.447 (0.548, 3.978)
Birth preparedness						
Yes	159	85.9	215	93.9	1	1
No	26	14.1	14	6.1	0.398 (0.201, 0.787)*	0.578 (0.257, 1.300)
Do you receive information on newborn care						
Yes	141	76.2	201	87.8	1	1
No	44	23.8	28	12.2	0.466 (0.265, 0.751)*	0.698 (0.389, 1.252)

* Reminded the significance of the variable (P value < 0.05)

In multivariate analysis, mothers’ age and occupation was found to be associated with the practice of newborn care; those respondents at the age 20–24 years old, the likelihood of good newborn practice was higher than those respondents at the age group 15–19 [AOR = 4.636 95% CI (1.024, 20.977)] and those respondents who were merchant was found 0.304 times less likely to have good practice towards newborn care than respondents who were housewife [AOR = 0.355 95% CI (0.133, 0.944)]. Respondents month of pregnancy at first ANC visit was found to be significantly associated with the practice of newborn care; those who started ANC visit during the second trimester 0.582 times less likely to have good practice than those started at the first trimester of pregnancy [AOR = 0.582 95% CI (0.352, 0.961)]. Knowledge and attitude on newborn care of the respondents were found to be significantly associated with their practice of newborn care; those respondents who had poor knowledge and negative attitude, were found 0.267 and 0.588 times less likely to have more good practice of newborn care than respondents with good knowledge and positive attitude [AOR = 0.267 (0.167, 0.428)] and [AOR = 0.588 (0.354, 0.977)] respectively (Table 3).

The article "Knowledge, practice and associated factors of newborn care among postnatal mothers at health centers, Bahir Dar City, Northwestern Ethiopia, 2016" was retracted in 2020. Reasons: plagiarism; content taken from a thesis; overlap with other authors' work.

**Table 3:** Association of knowledge on newborn care with socio-demographic and other factors, among postnatal mothers in Health Centers, Bahir Dar, Northwest Ethiopia, 2016 (N = 414)

Variable	Knowledge Level				Odds Ratio	
	Poor knowledge		Good knowledge		Crude	Adjusted
	N	%	N	%		
Age of mothers						
15–19	8	4.9	3	1.2	1	1
20–24	40	24.5	71	28.3	4.733 (1.188, 18.858)*	4.636 (1.024, 20.977)*
25–29	77	47.2	114	45.4	3.948 (1.015, 15.352)*	3.294 (0.745, 14.570)
30–34	27	16.6	49	19.5	4.840 (1.184, 19.775)*	4.544 (0.959, 21.545)
35–39	11	6.7	14	5.6	3.394 (0.725, 15.897)	5.912 (1.028, 33.978)
Maternal educational level						
No formal education	23	14.1	22	8.8	1	1
Read and write	10	6.1	19	7.6	1.986 (0.758, 5.205)	1.484 (0.435, 5.057)
Primary (1–4)	6	3.7	23	9.2	4.008 (1.372, 11.705)*	1.906 (0.543, 6.690)
Primary (5–8)	30	18.4	40	15.9	1.394 (0.657, 2.957)	0.506 (0.201, 1.276)
Secondary (9–12)	49	30.1	64	25.5	1.365 (0.683, 2.730)	0.486 (0.199, 1.185)
Tertiary (> 12)	45	27.6	83	33.1	1.928 (0.969, 3.837)	1.243 (0.467, 3.306)
Maternal monthly income						
151–650	55	33.7	98	39.0	1	1
651–1400	45	27.6	69	27.5	0.861 (0.522, 1.419)	0.706 (0.381, 1.310)
1401–2350	38	23.3	63	25.1	0.930 (0.553, 1.556)	0.612 (0.296, 1.2666)
2351–3550	20	12.3	15	6.0	0.421 (0.200, 0.888)*	0.355 (0.133, 0.944)*
3551–5000	5	3.1	6	2.4	0.673 (0.196, 2.308)	0.971 (0.212, 4.436)
Month of pregnancy at first ANC visit						
1–3 months	57	36.8	128	52.0	1	1
3–6 months	92	59.4	102	41.5	0.494 (0.324, 0 .752)*	0.582 (0.352, 0.961)*
6–9 months	6	3.9	16	6.5	1.187 (0.442, 3.192)	0.998 (0.265, 3.759)
No of ANC visits						
One	3	1.9	8	3.3	1.367 (0.353, 5.289)	2.311 (0.334, 15.965)
Two	14	9.0	15	6.1	0.549 (0.253, 1.192)	0.536 (0.195, 1.472)
Three	56	36.1	63	25.6	0.577 (0.368, 0.902)	0.633 (0.372, 1.079)
Four	82	52.9	160	65.0	1	1
Birth preparedness						
Yes	136	83.4	238	94.8	1	1
No	27	16.6	13	5.2	0.275 (0.137, 0.551)*	0.529 (0.213, 1.315)
Knowledge						
Poor knowledge	104	63.8	81	32.3	0.270 (0.179, 0.409)*	0.267 (0.267, 0.428)*
Good o knowledge	59	36.2	170	67.7	1	1
Attitude						
Negative attitude	63	47.0	71	53.0	0.626 (0.412, 0.951)*	0.588 (0.354, 0.977)
Positive attitude	100	35.7	180	64.3	1	1

* Reminded the significance of the variable (P value < 0.05)

### Discussion

In this study out of the total respondents interviewed, 229 (55.3%) of the respondents have good knowledge of newborn care and 251 (60.6%) of the respondents had a good practice. This figure is slightly higher than a study done in Madurai, Tamil Nadu India by which 61% of respondents had favorable attitude [8]. This discrepancy may be due to the fact that there is the socio-cultural difference. Also, the overall practice score of the study participants shows that majority 251 (60.6%) of the respondents had a good practice, which is higher than the finding of a study done in Mandura District, Northwest

Ethiopia, where (40.6%) of them had good newborn care practice [9]. This difference may be due to increased health services and great intervention focusing on child health.

The article "Knowledge, practice and associated factors of newborn care among postnatal mothers at health centers, Bahir Dar City, Northwestern Ethiopia, 2016" was retracted in 2020. Reasons: plagiarism; content taken from a thesis; overlap with other authors' work.

According to the result of the multivariate analysis, only mother ‘s level of education was significantly associated with their knowledge of newborn care at which respondents with primary [5–8] education and above were found to have more good knowledge about newborn care than those who had no formal education. This finding was similar with a study done in Tamil Nadu, in southeastern India and Kanchipuram district, India at which there was an association between knowledge and education [10, 11]. Similarly, educational status was significantly associated with the attitude towards newborn at which respondents with primary and above education are more likely to have a positive attitude towards newborn care than those who have had no formal education. Also, family monthly income and birth preparedness was significantly associated with their attitude towards newborn care.

Among those variables analyzed by multivariate analysis mothers ‘practice score had a significant association with mothers age, occupation, the month of pregnancy at first ANC visits, overall knowledge and attitude towards newborn care. Association of mothers occupation with practice finding was different from a study done in Mandura District, Northwest Ethiopia, in which no significant association between mothers occupation and newborn practice of the respondents [9]. This difference may be due to the difference in socio-demographic conditions in the study area.

Knowledge about newborn care association with the practices, which is in line with the finding of a study at Mandura District, Northwest Ethiopia, knowing first breastfeeding time and knowing first bathing time) were significantly associated with good newborn care practice of mothers [9].

## Conclusion

This study indicated that nearly half and above respondents had good knowledge and practice of newborn care and age of the mother, occupation, the month of pregnancy at first ANC visits, overall knowledge and attitude level was found to have a significant association with newborn care practice.

The article "Knowledge, practice and associated factors of newborn care among postnatal mothers at health centers, Bahir Dar City, Northwestern Ethiopia, 2016" was retracted in 2020. Reasons: plagiarism; content taken from a thesis; overlap with other authors' work.

## Limitation

Since this is a cross-sectional study, it may not show cause and effect relationship and small sample size.

## Data Availability

The data sets used and analyzed during the current study available from the corresponding author on reasonable request.

## Abbreviations

ANC: antenatal care
AOR: adjusted odds ratio
WHO: World Health Organization
SDG: sustainable development goal
SPSS: Statistical Package for Social Sciences
